This article has been retracted.

# Low back pain status in elite and semi-elite Australian football codes: a cross-sectional survey of football (soccer), Australian rules, rugby league, rugby union and non-athletic controls

**DOI:** 10.1186/1471-2474-10-38

**Published:** 2009-04-17

**Authors:** Wayne Hoskins, Henry Pollard, Chris Daff, Andrew Odell, Peter Garbutt, Andrew McHardy, Kate Hardy, George Dragasevic

**Affiliations:** 1 Division of Environmental and Life Sciences, Department of Health and Chiropractic, Macquarie University, NSW 2109, Australia; 2 Norwest Orthopaedic and Sports Physiotherapy, Norwest, NSW 2153, Australia; 3 Enhance Chiropractic and Massage Sports Injury Centre, Ngunnawal, ACT 2913, Australia

## Abstract

**Background:**

Our understanding of the effects of football code participation on low back pain (LBP) is limited. It is unclear whether LBP is more prevalent in athletic populations or differs between levels of competition. Thus it was the aim of this study to document and compare the prevalence, intensity, quality and frequency of LBP between elite and semi-elite male Australian football code participants and a non-athletic group.

**Methods:**

A cross-sectional survey of elite and semi-elite male Australian football code participants and a non-athletic group was performed. Participants completed a self-reported questionnaire incorporating the Quadruple Visual Analogue Scale (QVAS) and McGill Pain Questionnaire (short form) (MPQ-SF), along with additional questions adapted from an Australian epidemiological study. Respondents were 271 elite players (mean age 23.3, range 17–39), 360 semi-elite players (mean age 23.8, range 16–46) and 148 non-athletic controls (mean age 23.9, range 18–39).

**Results:**

Groups were matched for age (p = 0.42) and experienced the same age of first onset LBP (p = 0.40). A significant linear increase in LBP from the non-athletic group, to the semi-elite and elite groups for the QVAS and the MPQ-SF was evident (p < 0.001). Elite subjects were more likely to experience more frequent (daily or weekly OR 1.77, 95% CI 1.29–2.42) and severe LBP (discomforting and greater OR 1.75, 95% CI 1.29–2.38).

**Conclusion:**

Foolers in Australia have significantly more severe and frequent LBP than a non-athletic group and this escalates with level of competition.

## Background

The prevalence of low back pain (LBP) in the general population has been well described [1,2]. Despite most LBP being low-intensity and low-disability [3], figures documentetime prevalence have been as high as 84% with point-prevalence between 12% and 33% [2]. Less interest has been afforded to investigating LBP in athletic populations. In particular there are very few studies assessing LBP amongst active competing athletes, especially at the elite level of competition. Studies have documented that LBP prevalence and severity can vary between sports, with an increase in pain noted in those with significant low back demands [4,5]. Noteworthy is the reported lack of significant difference in low back injury rates between contact and non-contact sports [6].

It is not clear whether competing athletes are at a risk of a higher prevalence or increased intensity of LBP compared with the non-athletic population. It also has not been investigated whether LBP prevalence or intensity varies at different levels of athletic competition. Bahr et al [4]. analyzed LBP prevalence between elite athletes competing in endurance based sports: cross-country skiing (n = 257), rowing (n = 199), orienteering (n = 278) as well as a non-athletic group (n = 197). LBP lifetime (51–65%), year (48–63%) and 7 day prevalence (20–25%) was similar between groups although lower in non-athletes. No other large study has used homogeneity in study design and methodology to make direct comparisons between active athletes and non-athletes. Evidence suggests that sporting participation in the general population, regardless of activity, contributes to less frequent LBP [7]. However, once LBP is established, participation in sporting activities may indirectly contribute to increased severity of LBP [7]. Despite this, much of the current sporting literature has tended to focus on sports with specific low back demands such as rowing [4,8,9], skiing [4,10-12], gymnastics [13,14], wrestling [15], golf [16] and American football [17]. Less interest has been afforded to running based power sports.

The Australian football codes: football (soccer), Australian-Rules, rugby league and rugby union have established professional competitions. Each code has similar training and competition requirements, necessitating an all-round athletic ability with an emphasis on rapid acceleration running, endurance, agility, physical strength and code specific skills. Matches are played continuously over 90–120 minutes duration, typically weekly for the duration of the season.

The extent of LBP in elite Australian football code participants has not been fully elucidated. This could partly be the result of injury surveillance in Australian professional sport typically adopting an injury definition involving missed participation from a match [18-20]. Subsequently, the knowledge surrounding the prevalence and magnitude of LBP remains largely unknown. It is uncommon that LBP is severe enough to prevent a professional footballer from competing or from relinquishing his place in team selection. This is particularly true when medical management frequently incorporates epidural steroid injections [21] and local anaesthetic [22], considered 'part of the game' in professional football [23]. Despite this, injury surveillances have documented that low back injury if present can be severe and have high recurrence rates. In elite soccer, LBP is the most common overuse injury reported [24]. In elite rugby league, 'back injuries' have been shown to have the highest rates of recurrence for all injuries [25], whilst in retired elites chronic LBP is the third most common complaint, reported by 39% [26]. In elite Australian-Rules, 5% of players will miss a match each season with a 'lumbar or thoracic spine' injury, causing them to miss 4 weeks/matches [20]. In amateurs, 27% report a long term or recurrent back problem [27]. In school children playing rugby union, LBP afflicts over 40% of participants [28].

Our understanding of the effects of elite football code participation on LBP is limited. Thus, it was the objective of this study to determine the prevalence, intensity, quality and frequency of LBP in Australian football code participants. It was also our objective to compare this data between elite and semi-elite participants and with that of a non-athletic group.

## Methods

The study was designed as a cross-sectional survey of male Australian football code participants competing at the highest-level national or international elite competition (classified as elite), state based semi-elite competitions (classified as semi-elite) and a non-athletic control group (classified as non-athletic). The study was approved by the Macquarie University Human Ethics Committee.

Elite clubs were pragmatically selected to participate until an approximate equal percentage representation of total elite players from each code was achieved. For semi-elite participants, clubs were chosen from the various competitions within Australia until an approximate equal number of total players for each code was achieved. At both of levels of play, if clubs consented to participate it was required that they provide access to their entire player rosters to ensure 100% compliance which would assist in providing an accurate reflection of the status of LBP in the participating clubs. The survey commenced in early 2005. An attempt was made to standardise the time of delivery of the questionnaires. However, the scheduling of seasons of the codes and the different levels of play do not directly overlap. As such the questionnaires were completed at different times of the respective seasons but a feature was that all surveys were completed whilst in a period including either competition or pre-season matches. All athletes on the playing lists of the selected clubs were invited to participate and complete the survey with responses remaining confidential. Non-athletic controls were drawn from a convenience sample of age matched male University students and office workers, with the specification that they not participate in a football code at the elite or semi-elite level.

It should be noted that elite players are professional or 'full time' with their football commitments and this provides their sole income unless income is also received indirectly through their football requirements (e.g. endorsements). Semi-elite players receive financial payment but this is not enough to make them professional and they typically perform university study and/or work along with their football commitments to supplement their income.

The was presented to the clubs and players as a low back pain survey. Questionnaires were either administered by an author of the study or by an official representing the participating club, at the preference of the club. In the case of the club wishing to administer the survey, the questionnaires were mailed out along with consent forms and instructions describing the purposes and procedures of the study and how the instruments were to be administered. This was followed by a telephone call to confirm that all procedures would be correctly administered, to ensure players completed every question and to make certain the club officials were qualified to answer questions of the players. None of the assessors were involved in the analysis of the data. Analysis was provided by a person independent to each of the group allocations.

The questionnaire was developed using the validated and reliable Quadruple Visual Analogue Scale (QVAS) [29], the McGill Pain Questionnaire (short-form) (MPQ-SF) [30,31], along with a series of LBP questions either adapted from an Australian LBP epidemiological study with permission of the author [3] or that the authors developed themselves and thoroughly pilot tested.

The additional questions were:

• How old were you when you had your first ever attack or episode of LBP?

• If applicable, was this a result of your sporting commitments and activities or not related to this?

• When did your current episode of LBP commence?

• If applicable, was this a result of your sporting commitments and activities or not related to this?

• How often do you experience LBP?

To assist with answering the questions a diagram of a mannequin that defined the anatomical boundaries of the low back as a shaded area between the last ribs and the gluteal folds was provided (Figure 1). For the purposes of this survey the shaded area represented the low back and subjects were told to focus only on LBP and not other sources of pain. This area was found to be the most commonly used in a review of methodologically sound LBP prevalence studies [2].

**Figure 1:** **The anatomical boundaries representing the low back**.

The forms were manually entered using Microsoft Excel^® ^and analyzed using an Excel add-in (EcStat). The subject characteristics are reported as means, standard deviations and age range. One-way ANOVA's and Pearson's Chi squared analysis were used to determine differences between groups. Pearson's chi-squared statistic was used to test independence between categorical outcome and predictor variables. When this hypothesis was rejected, odds ratios were used to assess the strength and directions of the association. For non-binary variables the odds ratios provided are computed by comparing the odds of each specified outcome level for each given predictor level with reference categories obtained by aggregating those for all other levels. Odds ratios are reported with 95% confidence limits.

## Results

The subject characteristics of the different groups show groups were matched for age (Table 1). At the elite level 4 of the 14 (28.6%) Australian rugby league clubs (n = 93), 1 of the 2 (50.0%) rugby union clubs (n = 19), 3 of the 16 (18.8%) Australian-Rules clubs (n = 112) and 2 of the 6 (33.3%) soccer clubs (n = 47) participated. At the semi-elite level, 2 rugby league clubs participated (n = 52), 6 rugby union clubs (n = 139), 4 Australian-Rules clubs (n = 99) and 4 soccer clubs (n = 70). It appears that there was an almost linear trend of increasing LBP severity from the non-athletes, to the semi-elite and elite groups (Table 1). The elite athletes had significantly increased levels of the sensory, affective and total pain score when compared with both the semi-elite and non-athletic groups (Table 1). Elite athletes were approximately twice as likely to experience discomforting or greater LBP, less likely to have no LBP, whilst semi-elite athletes were less likely to experience discomforting or greater LBP and non-athletes more likely to experience no LBP (Chi squared χ^2 ^18.67, p < 0.001) (Table 2). Using the results of the question "what describes your overall LBP" from table 2, in terms of prevalence, the elite group has a figure of 77.9%, semi-elite 66.7%, and non-athletic 62.2%. When solely looking at those with discomforting or worse pain the figure for the elite group is 42.1%, semi-elite 29.7% and non-athletic 28.4%.

**Table 1:** Subject characteristics and results of the QVAS and MPQ-SF questionnaires by group (n = 779)

	**Elite**	**Semi-elite**	**Non-athletes**	**P value**
Number	271	360	148	
Mean age (SD)	23.3 (4.0)	23.6 (4.0)	23.9 (4.5)	0.42
Age range	17–39	16–46	18–39	
LBP now^a, b ^(SD)	25.4 (22.6)	17.7 (21.5)	11.2 (15.3)	<0.001
LBP average^a ^(SD)	24.9 (19.8)	19.4 (19.0)	11.2 (12.3)	<0.001
LBP best^a ^(SD)	8.5 (11.9)	5.2 (9.1)	2.3 (4.9)	<0.001
LBP worst^a ^(SD)	56.2 (27.6)	48.1 (28.6)	39.8 (25.3)	<0.001
Sensory pain score^b ^(SD)	16.5 (14.0)	12.8 (12.4)	9.8 (9.2)	<0.001
Affective pain score^b ^(SD)	8.4 (13.2)	6.9 (11.6)	5.6 (8.2)	0.047
Total pain score^b ^(SD)	14.3 (13.0)	12.2 (13.6)	9.3 (9.9)	<0.001

^a ^Questions from the QVAS

"LBP now" refers to the question: How much LBP do you have right now?

"LBP average" refers to the question: What is your typical or average pain?

"LBP best" refers to the question: What is your pain level at its best (How close to "0" does your pain get at its best)?

"LBP worst" refers to the question: What is your pain level at its worst (How close to "10" does your pain get at its worst)?

^b ^Questions from the MPQ-SF

**Table 2:** Self reported present LBP intensity by category (none, mild, discomforting) by group (n = 779)

**Level**	**Overall pain**^**a**^	**Odds ratio**	**95% CI**
Elite (n = 271)	None (n = 60, 22.1%)	0.54	0.38–0.75
	Mild (n = 97, 35.8%)	0.99	0.73–1.35
	Discomforting + (n = 114, 42.1%)	1.75	1.29–2.38
Semi-elite (n = 360)	None (n = 120, 33.3%)	1.31	0.96–1.77
	Mild (n = 133, 36.9%)	1.08	0.81–1.45
	Discomforting + (n = 107, 29.7%)	0.71	0.53–0.96
Non-athletic (n = 148)	None (n = 56, 37.8%)	1.53	1.05–2.22
	Mild (n = 50, 33.8%)	0.89	0.61–1.30
	Discomforting + (n = 42, 28.4%)	0.74	0.50–1.09

^a ^Question from MPQ-SF

Breakdown of discomforting, distressing and excruciating pain for the groups were elite (n = 88, 24, 2), semi-elite (n = 93, 8, 6) and non-athletic (n = 39, 2, 1) respectively. These levels of pain have been combined and are described as "discomforting +"

The results of the age of first ever episode of LBP were non-significant between groups (p = 0.40), with the means (SD): elites 17.9 (4.0), semi-elites 17.8 (4.0) and non-athletes 17.2 (4.1). Responders were 164 elites (60.5%), 220 semi-elites (61.1%) and 84 non-athletes (56.8%). Elite athletes were 2–5 times more likely to attribute their initial LBP to a sporting activity and less likely to be due to other factors (Table 3). Non-athletes experienced the opposite pattern whilst semi-elite athletes were also less likely to attribute sporting activity to initiate their first onset LBP (Chi squared χ^2 ^55.10, p < 0.001). Elite athletes were more likely to have a recent onset of LBP and less likely to not experience a current episode (χ^2 ^11.91, p = 0.018) (Table 3). Elite athletes were 2–4 times more likely to attribute sporting activity to have initiated their current LBP and less likely for other factors to be involved, whilst non-athletes report the opposite pattern, being 2–5 times more likely to attribute non-sporting factors to cause their LBP (χ^2 ^73.05, p < 0.001) (Table 3). Elite athletes were approximately twice as likely to report daily or weekly LBP and less likely to experience less-frequent LBP, whilst non-athletes report the opposite pattern, being approximately 2–3 times more likely to report fortnightly or less frequent LBP (χ^2 ^28.47, p < 0.001) (Table 3).

**Table 3:** LBP profile (pain association, onset and frequency) by group (n = 779)

**Level**	**Initial LBP due to sport**^**a**^	**Odds ratio**	**95% CI**
Elite (n = 271)	N/A (n = 13)	0.39	0.21–0.73
	Yes (n = 229)	3.40	2.34–4.94
	No (n = 29)	0.32	0.21–0.50
Semi-elite (n = 360)	N/A (n = 42)	1.78	1.08–2.92
	Yes (n = 235)	0.69	0.50–0.93
	No (n = 83)	1.21	0.86–1.71
Non-athletic (n = 148)	N/A (n = 16)	1.27	0.71–2.29
	Yes (n = 78)	0.40	0.28–0.58
	No (n = 54)	2.66	1.80–3.94

	**Start of current LBP episode**^**b**^		

Elite (n = 271)	N/A (n = 85)	0.58	0.43–0.80
	0–3 months (n = 110)	1.43	1.06–1.95
	>3 months (n = 76)	1.25	0.89–1.74
Semi-elite (n = 360)	N/A (n = 156)	1.34	1.01–1.79
	0–3 months (n = 117)	0.80	0.60–1.08
	>3 months (n = 87)	0.90	0.65–1.24
Non-athletic (n = 148)	N/A (n = 67)	1.34	0.93–1.92
	0–3 months (n = 47)	0.83	0.57–1.21
	>3 months (n = 34)	0.86	0.56–1.31

	**Current LBP due to sport**^**c**^		

Elite (n = 271)	N/A (n = 85)	0.61	0.45–0.83
	Yes (n = 173)	2.79	2.05–3.78
	No (n = 13)	0.22	0.12–0.41
Semi-elite (n = 360)	N/A (n = 151)	1.27	0.95–1.69
	Yes (n = 157)	0.75	0.56–0.99
	No (n = 52)	1.14	0.76–1.72
Non-athletic (n = 148)	N/A (n = 67)	1.38	0.96–1.99
	Yes (n = 40)	0.34	0.23–0.50
	No (n = 41)	3.34	2.14–5.19

	**Frequency of LBP**^d^		

Elite (n = 271)	N/A (n = 51)	0.84	0.58–1.22
	Daily or weekly (n = 107)	1.77	1.29–2.42
	Fortnightly + (n = 113)	0.68	0.50–0.91
Semi-elite (n = 360)	N/A (n = 84)	1.35	0.95–1.91
	Daily or weekly (n = 111)	0.96	0.71–1.30
	Fortnightly + (n = 165)	0.85	0.64–1.13
Non-athletic (n = 148)	N/A (n = 26)	0.78	0.49–1.25
	Daily or weekly (n = 26)	0.40	0.26–0.64
	Fortnightly + (n = 96)	2.34	1.62–3.40

^a ^Question: if applicable, was your first ever attack or episode of LBP a result of your sporting commitments and activities or not related to this?

N/A = I have not had a first ever attack or episode of LBP

^b ^Question: when did your current episode of LBP commence?

N/A = I do not have a current episode of LBP

^c ^Question: if applicable, is your current episode of LBP a result of your sporting commitments and activities or not related to this?

N/A = I do not have a current episode of LBP

^d ^Question: how often do you experience LBP?

N/A = I do not experience LBP

"Fortnightly +" relates to experiencing LBP on a fortnightly basis or less frequently

## Discussion

The main findings of this study were that Australian football code participants appear to experience LBP more frequently and severely than the non-athletic population. The difference was more evident in the elite group compared to the semi-elite group. We postulate that the higher intensive of play may be associated with the increased low back pain status. Of interest was the finding that elite, semi-elite and non-athletic groups all reported the same average age of first onset LBP although reported etiology differed.

Strengths of our study included the use of validated questionnaires to quantify the intensity (QVAS) and quality of LBP (MPQ-SF). This has not been performed previously when assessing athletic LBP sufferers. Functional disability associated with LBP was not determined. This important aspect was not investigated as it was felt that validated questionnaires in use to determine these parameters were not created for an elite athletic population and were likely to be irrelevant to their high-level functional demands, making comparisons vexed.

Limitations exist in the study conducted. Firstly, the convenience sample taken for the non-athletic population is not a random population sample and may not be representative. However, random sampling not producing a 100% response rate has been discussed as potentially leading to overestimates of LBP in similar research [4]. Our controls were used because of their likely non-elite or semi-elite athletic participation rate and likelihood to be matched for age. Additionally, football club selection was not random and may not be representative, although difficulty arrises in enticing professional clubs into research and it is likely that a random selection would have produced low response rates. As several of the elite competitions have grown in the number of participating clubs, we recommend that future studies consider broader club representation with a higher and more equal player representations from each sport.

Secondly, similar to Bahr et al. [2] our study was based on data from self-reported questionnaires and not more objective findings obtained from clinical interview, physical examination or advanced imaging. However, the QVAS and MPQ-SF have demonstrated validity and reliability. Nevertheless, it has been discussed that there may be potential difficulty in comparing the results between elite athletes and non-athletes. A well motivated athlete may under-report pain in order to improve performance, their chances of team selection and for a positive mind frame [32]. Alternatively, pain may be over-reported as it may be provoked easily by intense training and competition requirements and hinder athletic performance [32]. The athlete may therefore place a greater impact on pain. This situation is more of a concern as exaggeration of self-reported LBP and disability may be a predictor for LBP chronicity [33]. However, previous research on amateur athletes found psychosocial issues such as level of satisfaction with coaches or team-mates not to be related to the development of LBP [6]. Psychosocial factors may be more important for the professional elite athlete who has financial, contractual and performance concerns. In support of this, we found elite participants to have higher levels for the sensory, affective and total pain scores of the MPQ-SF, although we do not know why. Furthermore, it has been shown that LBP in former elite athletes is predicted by psychosocial issues such as life dissatisfaction, neuroticism, hostility, extroversion and poor sleep quality [34], whilst a recent prospective 5 year study of an employed group of participants has suggested that the vast majority of incident-adverse LBP events may be predicted not by structural findings or minor trauma but by a small set of demographic and behavioral variables [35]. Future research is required to more broadly investigate confounding variables including psychosocial factors in the elite athlete and their impact and relevance if any to the development of LBP during play and after a career has ended.

Thirdly, our study does not quantify what aspect of the Australian football codes is responsible for the increased frequency or severity of LBP. LBP could be related to the type, intensity, duration and/or amount of athletic activity performed. In endurance based sports with low back demands a dose response relationship appears to exist with LBP [4]. Further, whilst there is an increasing trend for reported first onset LBP to be a result of sporting commitments in football code participants, this may not necessarily be due to football code participation. At a young age, people tend to participate in multiple sports and activities. As some questions asked were retrospective in nature, there is likely an element of recall bias, which may have contributed to lower response rates when compared to the rates of questions requiring more recent recall.

It may be reasonable to conjecture that regardless of the etiology of the initial LBP, that once a footballer has experienced significant LBP, they remain susceptible to future pain and aggravation or exacerbation. This supports our findings that elite footballers were more likely to report a recent onset of LBP. Although likely to be multi-factorial, one explanation for recurrent LBP in athletes could be that athletes who demonstrate neuromuscular control alterations to sudden trunk loading have an increased risk of sustaining a low back injury [36]. Previously it has been shown that athletes with a recent acute low back injury exhibit altered neuromuscular control strategies for sudden trunk loading [37]. These findings are relevant to the contact Australian football codes but also for the agility, change of direction and sudden stop-start nature of all codes. Lumbar muscle activity during gait functions to control trunk movements [38]. In a non-athletic population, LBP was shown to produce poorly coordinated activity of the lumbar muscles during gait [39], which in a football player may lead to forces being directed at unprotected spinal structures producing subsequent mechanical stress and injury. Greater and more frequent mechanical spinal loading in elite footballers could contribute to both injury and delayed healing response. Similar to the non-athletic population, a situation may exist where LBP fluctuates over time with recurrences or exacerbations and temporary remissions [40,41]. Given footballers are exposed to greater and more frequent mechanical stresses in training and competition, this scenario appears likely. In support of this contention, Green et al. [6] documented that athletes with a history of low back injury with current LBP have a 6 times greater risk for future injury. For athletes with a previous history of low back injury approximately a 3 times greater risk of injury exists [6,36].

Low back injury in athletes may be of further significance as Nadler et al. [42] documented that athletes with resolved LBP from a history of low back injury demonstrate significantly diminished athletic performance in a 20 m shuttle run test compared with a healthy group. Further study is warranted in elite football code participants given the apparent scale of LBP and low back injury present. Future research is also required to document effective management strategies as apart from one short-term small study [43], we are not aware of randomized controlled trials for the treatment or rehabilitation of LBP with subjects drawn from an athletic population. The limitation in using current published evidence based guidelines for LBP management [44,45] is that acute pain advice generally advocates an approach to management that includes advice to: remain active, modify activity, remove only those activities that specifically aggravate and potential replace with other non aggravating activity (relative rest) and to stay at work. For chronic conditions various exercise-based protocols are often recommended. It may be for an athlete that the active approach and the tissue loading from many of the 'stabilization exercises' [46,47] they predictably already perform are etiological or aggravating or ineffective factors. In support of this assertion, there is no significant advantage of additional core-strengthening in reducing LBP occurrence in athletes [48]. It would be equitable to advocate that separate guidelines are required for the athletic population.

Questions need to be raised regarding whether LBP normalizes following a career of participation. It is known that former elite athletes are more likely to receive hospital care suffering from musculoskeletal complaints in general [49]. However, in the largest study performed using self-reported questionnaires, it appears that LBP is less common in former elite athletes (29.3% of 937) than in non-athletes (44% of 620) [34]. This is despite an increase in degenerative radiological findings in former elite athletes [32,34]. It is unclear whether participation in certain sports will affect post career pain or the intensity of LBP experienced [32].

## Conclusion

The main findings of this study were that elite football code participants in Australia compared with age-matched semi-elites and non-athletes have significantly higher levels and more frequent LBP and are more likely to attribute sporting activity as the etiological factor. Despite the age of onset of first time LBP being the same between groups the reported etiology differs. Predisposing factors need to be identified along with optimal methods of management for the athletic population of LBP sufferers given a current and a previous history of low back injury results in functional disturbances and may be detrimental to athletic performance and well-being in the short and long-term.

## Competing interests

The authors declare that they have no competing interests.

## Authors' contributions

HP and WH conceived the idea of the study. All authors were involved in recruitment of subjects and data entry. WH and HP contributed to writing an initial draft document. All authors contributed to the re-writing of this paper. All authors made original contributions to the content of the final manuscript. All of the authors participated in the editing and revisions of the multiple drafts that existed between the initial and final draft. All authors read and approved the final manuscript.

## Pre-publication history

The pre-publication history for this paper can be accessed here:


